# Overexpression of SATB1 Is Associated with Biologic Behavior in Human Renal Cell Carcinoma

This article has been retracted.

**DOI:** 10.1371/journal.pone.0097406

**Published:** 2014-05-16

**Authors:** Chao Cheng, Feng Wan, Lian Liu, Fuqing Zeng, Shi'an Xing, Xiaofei Wu, Xuepan Chen, Zhaohui Zhu

**Affiliations:** 1 Department of Urology, Union Hospital, Tongji Medical College, Huazhong University of Science and Technology, Wuhan, Hubei, China; 2 Cancer Center of Union Hospital, Tongji Medical College, Huazhong University of Science and Technology, Wuhan, Hubei, China; 3 Central Laboratory of Union Hospital, Tongji Medical College, Huazhong University of Science and Technology, Wuhan, Hubei, China; Cedars Sinai Medical Center, United States of America

## Abstract

Special AT-rich sequence-binding protein-1 (SATB1) has been reported to be aberrantly expressed in various cancers and correlated with the malignant behavior of cancer cells. However, the function of SATB1 in RCC remains unclear. With the combination of immunohistochemistry, western blotting, immunofluorescence, qRT-PCR, and cell proliferation, migration and invasion assays, we found that levels of SATB1 mRNA and protein were dramatically increased in human ccRCC tissues (P<0.001 for both), and upregulation of SATB1 was significantly associated with depth of invasion (P<0.001), lymph node status (P = 0.001) and TNM stage (P = 0.009). SATB1 knockdown inhibited the proliferation, migration and invasion of 786-O cells, whereas SATB1 overexpression promoted the growth and aggressive phenotype of ACHN cells *in vitro*. Furthermore, SATB1 expression was positively correlated with ZEB2 expression (P = 0.013), and inversely linked to levels of SATB2 and E-cadherin (P = 0.005 and P<0.001, respectively) in ccRCC tissues. Our data provide a basis for the concept that overexpression of SATB1 may play a critical role in the acquisition of an aggressive phenotype for RCC cells through EMT, providing new insights into the significance of SATB1 in invasion and metastasis of ccRCC, which may contribute to fully elucidating the exact mechanism of development and progression of RCC.

## Introduction

Renal cell carcinoma (RCC) is the most prevalent malignancy of the adult kidney, accounting for approximately 90–95% of all kidney neoplasms [1]. Worldwide, the incidence of RCC is over 200,000 new cases each year and mortality due to RCC has exceeded 100,000 annually [2], [3]. The clear cell renal cell carcinoma (ccRCC) is the most common histopathological subtype, comprising 70–80% of all RCCs [4]. Although considerable improvements have been made in diagnosis, surgical techniques and adjuvant therapies in last decades, patients with ccRCC still face a dismal clinical outcome owing to high rate of metastasis both at initial presentation and after radical nephrectomy [2], [5]–[7]. The overall five-year survival rate of patient with RCC ranges from 5% to 10%, with a median survival of only about 13 months [8], [9]. Therefore, it is of paramount importance to better understand the molecular mechanisms involved in the initiation and progression of RCC. Identification of novel biomarkers associated with disease progression and metastasis of RCC and combination of their application with traditional diagnostic and prognostic parameters would contribute to development of effective strategies for the prevention, early diagnosis and treatment of RCC.

Special AT-rich binding protein 1 (SATB1), the global chromatin organizer and transcription factor, is a cell type-specific nuclear matrix attachment region (MAR) DNA-binding protein and has the ability to participate in a variety of important biological processes including proliferation, differentiation, apoptosis, DNA recruit, transcription and reprogramming of expression profile [10]–[12]. SATB1 has a unique ‘cage-like’ protein distribution, which can provide docking sites for specialized DNA sequences and enzymes to control gene expression, including genes regulating cell adhesion molecules and EMT, by periodically anchoring matrix attachment regions to the nuclear matrix and directly recruiting chromatin remodeling complexes [13]–[16]. Therefore, SATB1 has been considered to be a new type of key gene regulator. Recently, increased expression of SATB1 has been found to be associated with invasion and metastasis of various types of cancers, such as breast cancer, gastric cancer, rectal cancer, liver cancer and prostate cancer, indicating the significance of SATB1 as an independent prognostic factor as well as a potential therapeutic target in human malignancies [12], [17]–[21].

However, SATB1 expression and its clinical significance in RCC remain unclear. In the present study, we immunohistochemically evaluated SATB1 expression in clinical ccRCC tissue specimens and determined its correlation with clinicopathological characteristics. Furthermore, SATB1 expression was detected in established human RCC cell lines including 786-O, A498 and ACHN to investigate the roles of SATB1 expression in biologic behavior of renal cancer cells by a combination of western blotting, quantitative real-time PCR, immunofluorescence staining, cell proliferation, migration and invasion assays.

## Materials and Methods

### Ethics statement

This study was performed under a protocol approved by the Ethics Committee of Union Hospital, Tongji Medical College, Huazhong University of Science and Technology (HUST), and written informed consent for participation in the study was obtained from each patient.

### Patients and tissue samples

A total of 89 pairs of ccRCC tissue samples and matched normal renal tissues were obtained from patients undergone surgical resection of primary ccRCC at Department of Urology of Union Hospital (Wuhan, China) between December 2010 and November 2012 for immunohistochemistry. The criteria for study enrollment were histopathological diagnosis of clear cell renal cell carcinoma, newly diagnosed and untreated, no history of other tumor, and the potential to follow up. The tumor stage and grade were recorded according to the tumor node metastasis staging system and Fuhrman criteria, respectively, in order to have a much better homogeneous comparison of present study to those in the literatures where the vast majority of the data adopted these staging and grading systems [2]. Clinical and pathologic information were collected from a retrospective review of well-documented medical records, and characteristics of patients were detailed in Table 1.

**Table 1:** Clinicohistopathologic characteristics of patients with ccRCC and their associations with SATB1 expression.

Characteristics	All cases	SATB1 expression		P-value
		High	Low	
Age (median 59)				0.351
≥59	46	17	29	
<59	43	24	19	
Gender				0.097
Male	57	30	27	
Female	32	11	21	
Tumor size				0.187
≤4.0	29	10	19	
4.1∼7.0	27	12	15	
>7.0	33	19	14	
Symptoms at diagnosis				0.053
Incidental	38	13	25	
Symptoms	51	28	23	
Depth of invasion				<0.001
T1+T2	51	16	35	
T3+T4	36	25	11	
Lymph node status				0.001
Negative	69	25	44	
Positive	20	16	4	
Distant metastasis				0.058
Absent	78	33	45	
Present	11	8	3	
TNM stage				0.009
I+II	66	25	41	
III+IV	23	16	7	
Fuhrman grade				0.355
G1-2	63	31	32	
G3-4	26	10	16	

### Immunohistochemistry and staining analysis

SATB1 expression was determined by immunohistochemical staining with the streptavidin biotin-peroxidase complex method using SABC kits (Boster Ltd., Wuhan, China) according to the manufacturer's protocol. In brief, formalin-fixed and paraffin embedded tissue sections (4 µm) were deparaffinized and rehydrated. Endogenous peroxidase activity was blocked with 0.3% hydrogen peroxide for 10 min. After antigen retrieval by microwaving, the slides were incubated with a rabbit polyclonal anti-SATB1 (1∶200; Abcam Inc., Cambridge, MA, USA) and anti-ZEB2 (1∶100; Sigma, St. Louis, MO, USA) in a humidified chamber overnight at 4°C, whereas anti-SATB2, anti-E-cadherin, anti-vimentin and anti-fibronectin (Santa Cruz Biotechnology Inc., Santa Cruz, CA, USA) were used at the dilution of 1∶100 for each. The streptavidin-peroxidase technique was used as described in our previous study [17]. Diaminobenzidine (DAB) was used as chromogen and the sections were counterstained with hematoxylin. Samples incubated with PBS instead of the primary antibody served as negative controls.

The immunohistochemical staining was randomly scored by two independent investigators in a blinded fashion, based on the intensity and percentage of cells with SATB1 staining. Referring to the predominant intensity, staining intensity was denoted as 0 (negative), 1 (weak), 2 (moderate) or 3 (strong). The score of staining density was given according to the percentage of positive staining cells as follows: 0, less than 5%; 1, 5 to 25%; 2, 25 to 50%; or 3, more than 50%. The final score was then calculated by adding the two above scores, and scores of 0–2 were considered as low expressions while scores of 3–6 were defined as high expressions [17], [22].

### Cell culture and transfection

Human RCC cell line 786-O and immortalized normal human proximal tubule epithelial cell line HK-2 were purchased from the American Type Culture Collection (ATCC, Rockville, MD, USA), and human RCC cell lines A498 and ACHN were purchased from the Cell Bank of Type Culture Collection of Chinese Academy of Sciences (Shanghai, China). All cell lines were preserved in our laboratory (Central Laboratory of Union Hospital, Tongji Medical College, HUST, Wuhan, China). HK-2 cells were cultured in K-SFM medium (Gibco Life Technologies, Grand Island, NY, USA), and other cells were cultured in RPMI-1640 medium supplemented with 10% fetal bovine serum and 100 µg/ml penicillin-streptomycin (Gibco, Carlsbad, CA, USA) under the conditions of 5% CO_2_ at 37°C. Cells were regularly passaged to maintain growing in the exponential phase. The SATB1 expression vector pcDNA3.1-SATB1 and SATB1-specific shRNA pGenesil2-SATB1 (the shRNA sequence was designed to target SATB1 as follows: 5′-GGAATGCTCTGAAGGACTTAC-3′) were constructed as described previously [19], and then transfected into 60%-confluent ACHN and 786-O RCC cells, respectively, using lipofectamin 2000 (Invitrogen, Carlsbad, CA, USA) according to the manufacturer's instructions. Following transfection, the transfected cells were allowed to recover for 24 h, and then individual clones with stable transfection screened with G418 (400 µg/ml) for two weeks were isolated. Thereafter, single colony of stable cells was picked and maintained in culture medium containing 200 µg/ml G418 to further culture. All the subsequent experiments were performed using the stable cells from single colony. Cells transfected with pcDNA3.1 or pGenesil2 control vector were used as negative controls.

### Cell migration and invasion assays *in vitro*

Transwell plates with 6.5 mm poly-carbonate filters and 8.0 µm pore size (Corning Costar, MD, USA) were used to determine the effect of SATB1 gene on migration and invasion of RCC cells. Cell invasion assays were performed in transfected cells (786-O and ACHN) according to previous described methods [23]. In brief, the transwell filter inserts were coated with 50 µl Matrigel (BD Biosciences, NJ, USA). An aliquot of 10^5^ cells were seeded into the upper chambers with 100 µl serum free medium, respectively, and the lower chambers were filled with medium contained 10% fetal bovine serum. After 24 hours incubation at 37°C in a 5% CO_2_ incubator, cells remaining on the upper chambers were gently removed with a cotton-tipped swab whereas the invasive cells attaching to the lower surface of the matrigel were fixed with 4% paraformaldehyde and stained with 0.1% Crystal Violet (Boster Ltd., Wuhan, China) according to the manufacturer's protocol. For quantification, the stained cells were counted under a light microscope in five fields (up, down, median, left, right; 200×). At least three chambers from three different experiments were analyzed statistically.

For migration assays, an aliquot of 10^5^ 786-O and ACHN cells were seeded in upper chambers without coated Matrigel. After 12 h incubation at 37°C, the cells had traversed the membrane were also counted and analyzed as described above.

### Cell proliferation assay

The cell growth rates were detected using a CCK-8 cell proliferation assay (CCK-8 kit; Boster Ltd., Wuhan, China) according to the manufacturer's instructions. In brief, the cells (4×10^3^/well) were seeded in a 96-well plate and cultured for 48 h at 37°C in a 5% CO_2_ atmosphere. After incubation with CCK-8 solution (10 µl/well) for 1 h, the absorbance value at 450 nm was measured using a microplate reader and analyzed at 24 h intervals [24], while the 650 nm served as the reference wavelength. All experiments were performed in triplicate, and the results were representative of three individual experiments.

### Immunofluorescence and confocal microscopy

Immunofluorescence staining with the antibody to SATB1 was performed to determine the expression and distribution of SATB1 in human RCC cell lines. Cells cultured on a 24-well plate were fixed in 4% paraformaldehyde for 20 min at 37°C, and then washed twice with PBS for 10 minutes. After permeabilized with 0.3% Triton for 15 minutes, cells were blocked with 5% BSA for 30 min. Subsequently, cells were incubated with a rabbit polyclonal anti-SATB1 (1∶200; Abcam Inc., Cambridge, MA, USA) overnight at 4°C, followed by visualization with a goat anti-rabbit IgG-TRITC (1∶100; Jackson, West Grove, PA, USA) for 1 hour at room temperature in the dark. Nuclei were stained with 4′, 6-diamidino-2-phenylindole (DAPI) for 5 min. Images were evaluated with a Nikon-A1Si confocal microscope (Nikon Corporation, Tokyo, Japan).

### Western blotting analysis

Western blotting was performed to determine SATB1 expression in human ccRCC tissues and cell lines. Briefly, total protein was extracted using RIPA Buffer (Sigma, St Louis, MO, USA), and protein concentrations were quantified by BCA Protein Assay Kit (Boster Ltd., Wuhan, China). Equal amounts of harvested protein samples were resolved on a 10% SDS–PAGE and transferred to PVDF membranes (Millipore Corporation, Billerica, MA, USA). The blotted membranes were blocked with 5% BSA in TBST for 2 h at room temperature, and incubated with the indicated primary antibodies overnight at 4°C. The rabbit polyclonal anti-SATB1 (Abcam Inc., Cambridge, CA, USA) was used at the dilution of 1∶1000, while GAPDH (Boster Ltd., Wuhan, China) was used as a loading control. The membranes were washed and then incubated with appropriate horseradish peroxidase (HRP)-conjugated secondary antibodies (Boster Ltd., Wuhan, China) for another 2 h at room temperature. Immunoblots were visualized by enhanced chemiluminescence using Supper Signal West Pico Trail Kit (Pierce Biotechnology, Rockford, IL, USA) according to the manufacturer's instructions.

### RNA extraction and quantitative real-time PCR assays

Total RNA was extracted and purified from frozen tissue samples and cell lines using the Trizol reagent (Invitrogen Corporation, Carlsbad, CA, USA) according to the manufacturer's instructions. cDNA was prepared as previously described and used as a template for quantitative real-time polymerase chain reaction (PCR) performed on an ABI StepOnePlus Real-Time PCR System using the SYBR Green Real-time PCR Master Mix (Applied Biosystems Inc., Foster City, CA, USA) [18]. The sequences of gene specific primers for SATB1 (forward, 5′-GTGGAAGCCTTGGGAATCC-3′; reverse, 5′-CTGACAGCTCTTCTTCTAGTT -3′) and GAPDH (forward, 5′-TCGGA GTCAACGGATTTGGTCGT-3′; reverse, 5′-TGCCATGGGTGGAATCATATTGGA- 3′) were designed using NCBI Primer-BLAST. The cycle threshold (Ct) values were standardized to Ct values of GAPDH, and fold difference in occupancy was calculated as follows: Fold difference = 2^−ΔΔCt^.

### Statistical analysis

The data were presented as mean±standard deviation (SD). Each experiment was repeated at least three times. The χ^2^ test or Fisher's exact test was used to analyze the associations between SATB1 expression and clinicopathological features of renal cancer. Significant differences between the groups were determined using the unpaired Student's *t*-test. All statistical tests were two-tailed and statistical significance was assumed for P<0.05. All statistical analyses were performed using SPSS 16.0 for Windows (SPSS Inc., Chicago, IL, USA).

## Results

### Expression of SATB1 increased in human primary ccRCC tissues and RCC cell lines

To investigate the expression and distribution of SATB1 protein and mRNA in ccRCC tissues, the immunohistochemistry, qRT-PCR and western blotting analysis were initially performed in 89 pairs of human ccRCC and matched normal tissues, respectively. SATB1 staining was shown mainly in the nuclei of cancer cells and a combination of the nucleus and cytoplasm, while positive signals were very rare in normal renal tissues (Fig. 1A). A significant upregulation of SATB1 protein was observed in the ccRCC tissues (P<0.001; Fig. 1B). To further confirm these observations, we investigated the expression of SATB1 in ccRCC tissues and paired tissues using western blotting. Our data clearly indicated that the cancer tissue had a drastic increase of SATB1 expression as compared with the corresponding normal tissues (Fig. 1C). In line with this, the expression of SATB1 mRNA was found significantly higher in ccRCC specimens than that in normal renal tissues (P<0.001; Fig. 1D).

**Figure 1:** Expressions of SATB1 in human ccRCC tissues and matched non-cancer tissues. **A**, immunohistochemical staining for SATB1 in representative sections. (**a**) Negative or low level staining of SATB1 in paired normal tissue; (**b**) Moderate staining of SATB1 in tumor tissue; (**c**) Strong staining in majority of ccRCC cells; (**d**) Negative control for SATB1 staining in ccRCC tissues. Magnification: 400×. **B**, The distribution of the difference in immunoreactivity score (IRS) of SATB1 staining. The IRS of SATB1 was obtained from 89 pairs of tissues, and the difference was expressed as ΔIRS = IRS_T_-IRS_N_ (T, tumor tissues; N, matched normal tissues). **C–D**, Expressions of SATB1 protein and mRNA in four representative pairs of matched normal renal tissues (N) and ccRCC tissues (T) were assessed by western blotting and qRT-PCR, respectively. Scale bar: 10 µM. Data were shown as mean ± SD (n = 3). **P<0.001.

In addition, the levels of SATB1 mRNA and protein were determined in four types of cell lines, including 786-O, A498, ACHN and HK-2. The expressions of both SATB1 mRNA and protein were significantly upregulated in RCC cell lines as compared with that in the immortalized normal human proximal tubule epithelial cell line HK-2 (Fig. 2A–B), which indicated SATB1 expression was associated with the aggressive phenotypes of RCC cells. Using the confocal microscopy, we found positive signals were predominantly localized in the nucleus with some amount of weak or moderate cytoplasmic staining (Figure 2C).

**Figure 2:** SATB1 expression is correlated with the aggressive phenotypes of renal cancer cell lines. SATB1 expression in immortalized normal human proximal tubule epithelial cell line HK-2 and three types of RCC cell lines (ACHN, 786-O and A498) was determined by qRT-PCR (**A**), western blotting (**B**) and immunofluorescent staining (**C**; Magnification: 200×), respectively. GAPDH served as a loading control. Scale bar represents 20 µM. Data were shown as mean ± SD (n = 3). **P<0.001.

### Immunohistochemical analysis of SATB1 expression in ccRCC clinical samples and its relationships to clinicopathological features

The relationships between SATB1 expression and clinicopathological parameters of ccRCC were summarized in Table 1. A total of 41 (46.1%) cases showed high levels of SATB1 expression (score 3–6). The increased expression of SATB1 protein showed a significant correlation with depth of invasion (P<0.001) and lymph node status (P = 0.001). Furthermore, our data also demonstrated that high SATB1 expression was dramatically associated with TNM stage (P = 0.009), which served as an important prognostic marker for patients with RCC. However, no significant association was found between SATB1 expression and other clinicopathologic features, including age, gender, primary tumor size, distant metastasis and Fuhrman grade.

### SATB1 depletion suppresses proliferation and aggressiveness of renal cancer cells *in vitro*

As shown in Fig. 2B, the 786-O cells had the highest level of SATB1 expression among the three types of renal cancer cell lines, and thus were selected for SATB1 gene silencing to study the effect of SATB1 knockdown on invasive phenotype and growth of renal cancer cells *in vitro*. After pGenesil2-SATB1-shRNA was transfected into 786-O cells, the level of SATB1 mRNA was remarkably reduced as compared with those transfected with control shRNA (P<0.001; Fig. 3A). Moreover, the expression of SATB1 protein was also significantly inhibited (P<0.001; Fig. 3B). These results indicated that SATB1 shRNA could effectively and specifically knockdown SATB1 expression at both transcriptional and translational levels.

**Figure 3:** Effects of suppression and overexpression of SATB1 on RCC cell line 786-O and ACHN. The 786-O cells were transfected with pGenesil2 control vector or pGenesil2-SATB1-shRNA, while ACHN cells were treated with pcDNA3.1 control vector or pcDNA3.1-SATB1, and nontransfected 786-O and ACHN cells were used as blank controls respectively. As compared to control groups, both mRNA and protein levels of SATB1were significantly decreased in 786-O cells after SATB1 knockdown (**A, B**), and remarkably increased in ACHN cells with SATB1 overexpression (**C, D**). Evaluation of cell proliferation by CCK-8 assays showed that down-regulation of SATB1 dramatically inhibited the cell proliferation rate of 786-O cells (**E**), whereas overexpression of SATB1 significantly promoted the growth of ACHN cells (**F**). Data were shown as mean ± SD (n = 3). *P<0.05, **P<0.001.

To further determine the effect of SATB1 on the migration, invasion and proliferation of renal cancer cells *in vitro*, the transwell migration and invasion assays and CCK-8 assay were carried out with 786-O cells, respectively. Our results showed that down-regulation of SATB1 in 786-O cells resulted in a significant inhibition of cell migration and invasion compared with that in the control shRNA-transfected cells (P<0.001; Fig. 4A–B). In CCK-8 assay, we observed that proliferation rate of cells treated with SATB1-specific shRNA was significantly decreased compared to cells transfected with control vector or parental cells (*P<0.05, **P<0.001; Fig. 3E). In summary, our data suggested that SATB1 expression obviously influences the proliferation, migration and invasion capacity of RCC cells.

**Figure 4:** Cell migration and invasion potential *in vitro* were evaluated by transwell migration and invasion assays. **A**, Silencing of SATB1 inhibited the cell migration and invasion capability of 786-O cells. **B**, Quantitative analysis of the number of 786-O cells that successfully migrated and invaded. **C**, SATB1 overexpression promoted the migration and invasion of ACHN cells. **D**, The number of migrated and invaded ACHN cells increased with SATB1 upregulation. Scale bar: 10 µM. Data were shown as mean ± SD (n = 3). **P<0.001. Magnification: 200×.

### Overexpression of SATB1 augments the growth and aggressive phenotype of renal cancer cells *in vitro*

We next examined whether ectopic expression of SATB1 was sufficient to promote the growth, migration and invasion capability of human renal cancer cells. After pcDNA3.1-SATB1 was stably transfected into the ACHN cells in which SATB1 expression was relatively low, both the mRNA and protein levels of SATB1 were dramatically up-regulated as compared with those in the nontransfected group (P<0.001; Fig. 3C–D), Furthermore, the migration and invasion capability was significantly increased to approximately 4.0- and 3.7-fold *in vitro* (P<0.001; Fig. 4C-D), respectively. However, no significant difference was observed between the pcDNA3.1 empty vector-transfected group and the control group. These data confirmed that ectopic expression of SATB1 in ACHN cells by pcDNA3.1-SATB1 vector could promote their capability of migration and invasion.

Additionally, we employed the CCK-8 cell proliferation assay to test effects of SATB1 overexpression on cell growth of ACHN. As compared with control cells and cells transfected with pcDNA3.1 empty vector, the pcDNA3.1-SATB1-transfected cells showed a greater proliferation ratio and higher relative absorbance value (*P<0.05, **P<0.001; Fig. 3F). Taken together, these results suggested that overexpression of SATB1 could facilitate the growth and aggressive phenotype of renal cancer cells *in vitro*.

### Expressions of EMT markers and SATB2 in ccRCC tissues and their correlations with SATB1 expression

To investigate the phenomenon and mechanism of SATB1-mediated regulation on invasive and metastatic capacity of ccRCC, additional immunohistochemical staining were utilized to detect the levels of EMT markers (including E-cadherin, ZEB2, vimentin and fibronectin) and SATB2, a homologue of SATB1, and analyze the potential correlations between SATB1 and expressions of EMT markers or SATB2 in ccRCC tissues. We found that SATB1 and ZEB2 levels were significantly up-regulated in ccRCC tissues as compared with those in the paired normal tissues, whereas the expressions of SATB2 and E-cadherin were remarkably decreased in cancer tissues (Fig. 5). Further correlation analysis revealed that the high level of SATB1 expression was positively correlated with ZEB2 expression (P = 0.013; Table 2). Moreover, significant inverse correlations were observed between SATB1 level and expressions of SATB2 and E-cadherin proteins, respectively (P = 0.005 and P<0.001, respectively; Table 2). However, no significant correlation was found between SATB1 expression and expressions of vimentin and fibronectin proteins (P>0.05 for both; Table 2).

**Figure 5:** Correlations between SATB1 and EMT markers or SATB2 in ccRCC tissues and paired control tissues. Negative SATB1 staining (**A**) and high expressions of SATB2 (**C**) and E-cadherin (**E**) were shown in matched normal renal tissues, respectively. Positive SATB1 staining (**B**) and high ZEB2 expression (**D**) were observed in ccRCC tissues. (**F**) Negative control in ccRCC tissues. (Hematoxylin counterstain; Magnification: 400×). Scale bar: 10 µM.

**Table 2:** Correlations between SATB1 level and expressions of SATB2 and EMT markers in ccRCC tissues.

Variable		SATB1 expression		R-value	P-value
	Cases	High	Low		
ZEB2 expression				0.262	0.013
High	46	27	19		
Low	43	14	29		
E-cadherin expression				−0.427	<0.001
High	40	9	31		
Low	49	32	17		
Vimentin expression				0.131	0.223
High	33	18	15		
Low	56	23	33		
Fibronectin expression				−0.193	0.071
High	44	16	28		
Low	45	25	20		
SATB2 expression				−0.296	0.005
High	38	11	27		
Low	51	30	21		

## Discussion

In the current study, we provided evidence for the first time that SATB1 was overexpressed mainly with a nuclear pattern in human clear cell renal cell cancer specimens, which was significantly associated with aggressive phenotypes of tumor cells. In keeping with these findings, our data further revealed that depletion of SATB1 suppressed the proliferation and aggressiveness of renal cancer cells with higher invasive activities *in vitro*; on the contrary, ectopic introduction of SATB1 resulted in increased growth and aggressive phenotype of renal cancer cells, which was probably due to induction of EMT *in vitro*. These results suggest that SATB1 is crucially implicated in the carcinogenesis and invasion of human renal cancer.

As a global chromatin organizer and transcription factor, SATB1 plays critical roles in integrating higher-order chromatin architecture with gene regulation [16]. In recent years, increasing bodies of researches have mainly focused on the correlations between SATB1 expression and the development and progression of several human solid tumors, and roles of SATB1 in a variety of cancer cells have been widely documented. Han *et al* reported that overexpression of SATB1 was significantly associated with both tumor invasive behavior and metastatic phenotype in breast cancer, and thus SATB1 protein had been proposed as a novel biological marker for breast cancer progression and metastasis [12]. Besides breast cancer, aberrant expression of SATB1 was also correlated with advanced clinicopathologic factors and poor prognosis in cases of glioma, melanoma and carcinomas of stomach, rectum, liver, bladder, and prostate [17]–[21], [25]–[27]. These results correspond well with our present findings, which provided additional evidence for the concept that SATB1 plays a crucial role in promoting tumor growth, invasion and metastasis of various types of malignancies, and may also have a potential value of being a molecular target for cancer therapy.

In order to provide further support that SATB1 contributes to the development and progression of renal cancer, several RCC cell lines (786-O, A498 and ACHN) were employed for gain and loss of function experiments. In light of our results, the levels of SATB1 in 786-O cells and ACHN cells were the highest and the lowest, respectively. Based on these findings, we effectively down-regulated SATB1 expression in 786-O cells by pGenesil2-SATB1-shRNA *in vitro*, and our data indicated that proliferation and invasiveness of stable transfected cells were significantly decreased. On the contrary, overexpression of SATB1 in ACHN cells mediated by pcDNA3.1-SATB1 resulted in the increased growth and aggressive phenotype *in vitro*. Taken together, both gain and loss of function experiments further confirmed that upregulation of SATB1 could facilitate the proliferation and aggressiveness of renal cancer cell lines *in vitro*, which was consistent with our data from the immunohistochemical analysis using the clinical ccRCC samples.

SATB1 is a cell type-specific nuclear MAR DNA-binding protein, which is 763 amino acids in length and is located on chromosome 3p23. Recently, SATB1 has attracted considerable attention due to its capability to coordinate regulation for many genes which are significantly associated with the growth, invasion and metastasis of a variety of malignancies [14], [15], indicating this “genome organizer” may have a crucial role in the complex gene expression patterns of human cancers by many mechanisms [26], [28]. A recent study by Tu *et al*. using the expression microarray analysis demonstrated that SATB1 could regulate expressions of over 100 genes related to tumor growth and metastasis [19]. SATB1 could upregulate the expressions of many genes which had critical roles in promoting tumor growth and metastasis (e.g. cell cycle progression-promoting gene CDK4, MMPs, Snail1and Slug), while many tumor suppressor genes (e.g. cell cycle arrest factors p16^INK4A^, promoting apoptosis gene FADD and epithelial markers E-cadherin) were significantly downregulated [19]. In addition, Han *et al* examined expression of SATB1 in breast cancer cells by gene expression profiling, and described that knockdown of SATB1 mediated by specific RNA-interference in highly aggressive (MDA-MB-231) cancer cells significantly changed expression levels of over 1,000 genes, resulting in tumorigenesis reverse and growth and metastasis inhibition of breast tumor *in vivo*, and most of these genes were associated with cell adhesion, phosphatidylinositol signaling and cell cycle regulation [12]. As an adherens junction protein and tumor suppressor, E-cadherin is commonly lost in invasive tumors which is a central event in the epithelial to mesenschymal transition (EMT) [29]. According to the findings reported by Han *et al*, E-cadherin was downregulated by aberrant expression of SATB1, whereas SATB1 depletion could upregulate E-cadherin expression and reverse EMT process, resulting in the restoration of acinar-like morphology [12]. Additionally, some of studies have thoroughly revealed the important role of ZEB2 expression in repression of E-cadherin [30], [31]. Therefore, we speculate that upregulation of SATB1 may contribute to the initialization of EMT process during the invasion and metastasis of RCC, which may explain our observation that SATB1 expression was dramatically associated with invasion and lymph node metastasis of ccRCC and that SATB1 expression was positively correlated with ZEB2 expression and inversely correlated with the level of E-cadherin in our ccRCC cohort, respectively. Combined analysis of SATB1 and EMT markers expressions may have significant values in determining invasion and metastasis and assessing prognosis of ccRCC, and SATB1 might also have a potential value of being a good molecular target for ccRCC therapy.

Our findings provide evidence for the emerging links among SATB1, expressions of EMT markers and tumor progression; however, there were some limitations in the current study. For instance, the *in vivo* assays should be performed to further testify the roles of SATB1 in progression and metastasis of human ccRCC, and the prognostic significance of high SATB1 expression for patients with ccRCC also need to be determined in future. Moreover, whether SATB1 directly binds to the MARs of EMT markers (e.g. ZEB2 and E-cadherin) to alter their expressions or indirectly regulates their expression through other signaling pathways are still required to be fully elucidated in the further investigations.

In summary, our data provided a basis for the concept that SATB1 expression was significantly upregulated in ccRCC tissues and RCC cell lines, which might be associated with adverse biologic behavior of cancer cells to promote the tumorigenesis and progression of RCC. More importantly, significant correlations between SATB1 expression and EMT markers were observed in the present study. Work is in progress in our laboratory to target the specific mechanisms by which SATB1 promotes tumor metastasis and correlate these findings with the overall survival rate of patients with ccRCC. The latter may be potentially significant to suggest that targeting of the SATB1 pathway may constitute a novel treatment modality for the prevention of ccRCC progression.

## Supporting Information

Figure S1 **Representative patterns of immunohistochemical staining for SATB2 (A, C) and E-cadherin (B, D) in human ccRCC tissues and paired non-cancerous tissues.** Both SATB2 and E-cadherin levels were significantly down-regulated in ccRCC tissues(A, B) as compared with the corresponding normal kidney tissues (C, D) (Magnification: 400×).
(TIFF)
